The article "Medical Communication Services after Traumatic Spinal Cord Injury" was retracted in 2023. Reasons: signs of a paper mill; suspected computer-generated content; unreliable results or conclusions; concerns about the data.

# Medical Communication Services after Traumatic Spinal Cord Injury

**DOI:** 10.1155/2021/4798927

**Published:** 2021-08-31

**Authors:** Jamal Alshorman, Yulong Wang, Fengzhao Zhu, Lian Zeng, Kaifang Chen, Sheng Yao, Xirui Jing, Yanzhen Qu, Tingfang Sun, Xiaodong Guo

**Affiliations:** Department of Orthopedics, Union Hospital, Tongji Medical College, Huazhong University of Science and Technology, Wuhan 430022, China

## Abstract

It is difficult to assess and monitor the spinal cord injury (SCI) because of its pathophysiology after injury, with different degrees of prognosis and various treatment methods, including laminectomy, durotomy, and myelotomy. Medical communication services with different factors such as time of surgical intervention, procedure choice, spinal cord perfusion pressure (SCPP), and intraspinal pressure (ISP) contribute a significant role in improving neurological outcomes. This review aims to show the benefits of communication services and factors such as ISP, SCPP, and surgical intervention time in order to achieve positive long-term outcomes after an appropriate treatment method in SCI patients. The SCPP was found between 90 and 100 mmHg for the best outcome, MAP was found between 110 and 130 mmHg, and mean ISP is ≤20 mmHg after injury. Laminectomy alone cannot reduce the pressure between the dura and swollen cord. Durotomy and duroplasty considered as treatment choices after severe traumatic spinal cord injury (TSCI).

## 1. Introduction

Most sufferers of complete SCI are paralyzed, with no bladder, bowel, or sexual function [1]. The swollen spinal cord is compressed by the dura mater, leading to raised intraspinal pressure (ISP). The worse the cord perfusion, the worse the prognosis [2, 3]. Current research has shown that the optimal spinal perfusion pressure (SCPPopt) varies from person to person [4], and no factor accurately predicts SCPPopt. It is important to monitor SCPPopt through pressure measurement and individual targeted perfusion [5]. The treatment method can then be adjusted to improve blood perfusion and prognosis and to prevent secondary injury [6, 7]. Maintaining mean arterial pressure (MAP) at 85–90 mmHg up to one week can be helpful in obtaining acceptable SCPP.

An appropriate treatment method is necessary to reduce ISP and achieve significant outcomes. However, there is no literature on how myelotomy can improve ISP. Performing bony decompression is not enough to decrease the pressure around the cord. Even if bony decompression is performed early, gradual or immediate swelling can cause subarachnoid occlusion [8]. The response depends on the initial severity of the injury; these points need a treatment that is effective in reducing swelling to optimize the clinical outcome [9]. This review aims to present different factors that affect the prognosis in SCI patients and compare the effect of myelotomy and durotomy procedures in humans and animals with SCI.

The article "Medical Communication Services after Traumatic Spinal Cord Injury" was retracted in 2023. Reasons: signs of a paper mill; suspected computer-generated content; unreliable results or conclusions; concerns about the data.

## 2. Material and Methods

Between April and October 2020, the authors collected articles through PubMed, Web of Science, and Google Scholar using different keywords combinations: durotomy, myelotomy, ISP, SCPP, SCI. Morover, the factors affect the prognosis after SCI with hemorrhage or edema in humans and animal experiments were collected. We then pared down the list of keywords based on relevance to the issue of SCI treatment and the best way to decrease ISP and increase blood perfusion at the injury site. Articles published from 1976 to 2020 were used to conduct our review.

### 2.1. Inclusion and Exclusion Criteria

Randomized SCI articles were added, including original articles, case reports, and animal studies. Acute and chronic injuries were included. Cervical, thoracic, and lumbar region that reported different procedures (durotomy and myelotomy) and the effect of these methods in achieving good or bad outcomes were studied. Monitoring ISP and SCPP provides information about prognosis and improve the neurological outcome [10]. We did not exclude studies based on patient characteristics, the timing of outcome assessment, study design, language, or publication status.

### 2.2. Statistical Analysis

Patients and animals data were analyzed using SPSS statistical software (IBM version 22). Different procedures were compared along with the improvement in neurological symptoms. The *P* value was 0.05.

## 3. Result

Thirty-seven articles were collected. Thirteen articles were of animal models (Table 1), and 24 were clinical studies, including nine case reports (Table 2). Four hundred seventy-nine animals were included in nine articles, and 34.2% used myelotomy as the procedure, including 6.2% that supported its use as a safe procedure and 12.4% that did not support it. Additionally, 6.2% supported myelotomy in the anteroposterior plane, which can show significant improvement but not in the dorsal midline. Thirty-eight percent support the use of durotomy, which can achieve better outcomes and help decrease ISP; 7.4% supported the addition of duroplasty to durotomy, and 18.5% mentioned that laminectomy alone cannot reduce ISP.

Of the twenty-three clinical articles, which included 523 patients, 37.2% described the use of durotomy and suggested it as the treatment of choice in SCI patients. Of the clinical cases, 16.7% suggested the use of durotomy with duroplasty for better prognosis, and 0.4% used laminectomy alone. Of the clinical cases, 4.1% concluded that durotomy and myelotomy are safe, and 56.7% of patients underwent ISP and SCPP monitoring. Of the patients, 4.3% showed that lumbar CSF drainage does not help reduce ISP and does not improve prognosis, and 1.6% used a different technique to treat SCI. Two clinical articles support myelotomy as a treatment procedure with good outcome.

The article "Medical Communication Services after Traumatic Spinal Cord Injury" was retracted in 2023. Reasons: signs of a paper mill; suspected computer-generated content; unreliable results or conclusions; concerns about the data.

### 3.1. Clinical Studies

A case report by Dickerman et al. treated by durotomy showed full recovery after eight weeks; CSF leakage was not detected [11]. Furthermore, Perkins and Deane observed six cases that underwent durotomy, half of whom recovered fully, whereas the other half recovered only partially [3]. Essentially, all patients showed functional recovery. Phang et al. introduced a case of eleven patients who were treated by laminectomy alone [12–14]. In contrast, he studied the results of another ten patients who underwent duroplasty in addition to laminectomy. Although the procedure (durotomy) can cause CSF leakage and pseudomeningocele, five patients were found to have undergone complete recovery. Thus, he concluded that adding duroplasty to the laminectomy procedure yields greater improvement than laminectomy alone. A study conducted by Xie et al. observed sixteen grade B patients, thirteen grade C patients, and six grade D patients [15]. Three months after the durotomy, patients' motor score, light touch score, and pin prick score increased significantly. Grassner et al. treated a man with durotomy but intraoperatively; the ISP increased at the injury site and during the post one-year follow-up, the patient showed no change in his neurological status [8]. Lee et al. examined a 47-year-old woman treated by the decopression method of thoracic ossification of the posterior longitudinal ligament, and MRI revealed CSF collection and spinal cord compression [16]. She was treated using double-layer duroplasty to prevent CSF leakage. A clinical study of seventeen patients by Telemacque et al. with ten patients without durotomy and seven patients with durotomy revealed that six of them showed positive prognosis [17]. Specifically, one patient showed improvement from ASIA grade A to grade C and another one from A to D. Furthermore, two patients of ASIA grade B improved to grade D, two patients from grade C to grade D, and one remained grade C. Qu et al. [18] conducted a study of 21 cases with or without hemorrhage who were treated by durotomy or myelotomy. Hui et al. performed durotomy to restore CSF flow and removed necrotic tissue, which showed good improvement in all the patients [19]. Moreover, rehabilitation for three months after the surgical intervention of 17 days can improve motosensory functions. Among ten grade B ASIA patients, seven improved to grade C, 2 to grade D, and one to grade E. Among 5 patients of grade C, four became grade D and one grade E. Six patients of grade A remained the same but showed some improvements in feeling and movements. Ramos et al. present two cases of spinal stenosis who underwent laminectomy and developed epidural abscess; after evacuating abscess, both patients showed good recovery [20]. Esfahani et al. presented a case report of a 60-year-old man laminectomy performed to treat L4 fracture; no hematoma was encountered, but after using ultrasound intraoperatively, a hematoma was detected and removed by durotomy; luckily, patient ASIA grade improved from D to E [21]. Ge et al. used ultrasound intraoperatively for a 68-year-old man complaining of lower back pain because of herniated disc, but ultrasound showed a mass that was treated by durotomy and he became normal after three months [12]. Koyanagi et al. presented four cases with good prognosis after myelotomy, but all the cases were acute SCI [22]. A 55-year-old woman treated by durotomy and duroplasty by Roy et al. revealed chronic spinal cord compression after MRI, but the patient made good recovery after the operation [23]. A 76-year-old man was treated by laminectomy and discectomy, but on the second day after the operation, he showed negative prognosis, and MRI demonstrated subdural fluid collection that was evacuated by durotomy and the patient went to a full recovery [24]. A study conducted by Saadoun et al. on 45 patients who underwent laminectomy with durotomy and duroplasty showed that durotomy with duroplasty can help in reducing ISP and increasing SCPP, leading to a better prognosis [25].

The article "Medical Communication Services after Traumatic Spinal Cord Injury" was retracted in 2023. Reasons: signs of a paper mill; suspected computer-generated content; unreliable results or conclusions; concerns about the data.

Werndle et al. developed a novel technique (pressure probe placed subdurally) to monitor ISP after chronic SCI in 18 patients with ASIA (A-C) grades [26]. They found that continuous measuring of ISP at the injury site is a safe procedure after TSCI. They inserted a pressure probe intradurally in 42 patients (ASIA grade A-C) with severe TSCI, treated by laminectomy [27]. Monitoring started 72 hours after the injury and continued up to one week; CSF leakage was found in three patients and pseudomeningocele in 8 patients, which resolved after six months of follow-up. Phang et al. placed pressure probe and microdialysis catheter at the injury site in 14 patients without any severe complication [28]. They aimed to optimize the SCPP at the injury site and recommended maintaining MAP at 85 to 90 mm Hg for a week after SCI. Layer et al. inserted a scaffold device 9 to 83 hours after injury in eight patients injured in the thoracic region, four patients improved to AISA grade B, one patient improved to grade C, and three patients remained grade A without any improvements [29]. A study predicted clinical factors in 64 patients (ASIA grades A–C) instead of ISP monitoring [5]. They found that reducing surgical bleeding and performing duroplasty can reduce ISP, but no factor predicted with SCPP. Association Impairment Scale A-C in 15 SCI patients received a lumbar subarachnoid drain (LSAD) by Yue et al. to monitor SCPP for five days and SCPP of ≥65 mm Hg in all patients with no complications [30]. Werndle et al. recommended to develop a method to measure the intrathecal pressure at injury site, to perform durotomy with duroplasty, and repeat MRI to evaluate the effect of treatment and recommended to focus more on the cord perfusion, preventing secondary injury [31]. The lumbar intrathecal catheter was inserted for 72 hours in 22 patients divided into two groups to drainage or nondrainage CSF to reduce the pressure after acute TSCI, and Kwon et al. reported that CSF drainage was not very helpful. During the first week after injury, MAP and CSF pressure were monitored in acute SCI patients (*n* = 92) by Squair et al. [32] to calculate SCPP [33]. Perfusion pressure lower than 50 mm Hg showed less neurological improvement. Gallagher et al. collected 22 patients and used laser speckle contrast imaging intraoperatively to visualize blood flow at the injury site. In acute and chronic SCI patients, they found three blood flow patterns (necrosis penumbra, hyperperfusion, and patchy perfusion) [34]. They concluded that interventions to increase pressure might increase spinal cord blood flow.

The article "Medical Communication Services after Traumatic Spinal Cord Injury" was retracted in 2023. Reasons: signs of a paper mill; suspected computer-generated content; unreliable results or conclusions; concerns about the data.

### 3.2. Animal Studies

Khaing et al. claimed that using microcatheter can allow for direct measurement of ISP after spinal cord injury and increasing tissue pressure can prevent better prognosis post-SCI [2]. A study concluded that duroplasty following acute SCI can reduce the meningeal fibrosis through increasing CSF flow at injury site and decrease inflammatory process around the injured cord. However, improving the CSF circulation can allow for better recovery by increasing the waste clearance system [35]. Seventy-two rats were assigned into three groups by Smith et al., and the rats treated with decompression and duroplasty showed better neurological recovery after acute cervical SCI compared with those treated only by decompression method [36]. A 15 spinal cord section from pigs was presented, and the pressure was different according to individual pig and the anatomic level; also it was concluded that durotomy can decrease the elevated pressure [37]. Zhang et al. compared three group of rats and BBB (Basso, Beattie, Bresnahan) score was used to evaluate the ability of rats; they suggested that longitudinal durotomy can improve the recovery in SCI rat model [38]. If the influence force is mild, and the hematoma is little or absent, more spared tissue nearby the lesion will be protected. Removing the hemorrhagic tissue by myelotomy may induce additional destruction to the normal tissue. Yang et al. mentioned that if a durotomy was applied as a control, then conclusion would be more powerful [39]. In addition, Iwasaki et al. presented two groups of dogs by performing myelotomy with or without steroid injection, in which both groups revealed the same outcome and did not show good prognosis [40]. An experiment study of 40 rats by Rivlin and Tator showed significant improvement only after performing anteroposterior myelotomy, but Dorsal midline myelotomy did not show any improvement [41]. Meyer et al. performed myelotomy on 20 rats, which reduced the BBB score and has no advantages [42]. But other study concluded the benefit of using myelotomy as a treatment procedure in 20 rats, and it improved the motor functions and reduced the edema [43]. Laminectomy plus cord incision showed better outcomes during the postoperation period, which started at 7 days postoperation [44]. Adding duroplasty to durotomy can reduce inflammation and scar formation. Moreover, a significant decrease in cavitation [36] presenting the edema and hematoma in big size after the injury prevent the CSF circulation, so evacuating the hematoma can recirculate the CSF and avoid further inflammation.

The article "Medical Communication Services after Traumatic Spinal Cord Injury" was retracted in 2023. Reasons: signs of a paper mill; suspected computer-generated content; unreliable results or conclusions; concerns about the data.

Jones et al. used ultrasound to visualize the dura and subrachnoid in 13 pigs with SCI; they reported that decompression after acute SCI may cause gradual or immediate swelling and subarachnoid occlusion [9]. These findings may partly describe the absence of the advantage of decompression in some patients and emphasize the importance of decreasing cord swelling to optimize the clinical result following acute SCI.

Secondary injury affects blood circulation, causing a further inflammatory response and local changes that contribute to additional neurological damage [45]. Injured area takes three forms (above, injury site, and below), ISP varies depending on the form and anatomical level [14]. Monitoring ISP is essential to predicting prognosis, but measuring via lumbar CSF catheter is insufficient [33, 46]. It is feasible to monitor ISP using a Codman device positioned at the location of the maximum swelling of the spinal cord as measured by MRI. CT scan can be used to determine the appropriate place of the probe [47].

### 3.3. Aging and the Effect on SCI

Age of the patients matter a lot especially in patients with osteoporosis because the bone density is less and the fracture will be more severe. Moreover, the patients are at higher risk of bone fragment, which may affect the dura and cause CSF leak out and increase the injury complications and worse the prognosis with poor outcomes. As the person gets old, the vessels wall can lose its elastic characteristic and can make poor blood perfusion compared with younger patients; so performing durotomy and duroplasty can give better environment for best recovery. Vascular factors and aging may increase the perfusion pressure around the cord and MAP, which can increase the resistance and decrease blood flow [48]. Presence of cardiovascular disease can affect the blood circulation, which make blood flow to the injury site harder and delay the prognosis. Using some drugs (heparin, and vitamin K antagonists) for long time can decrease the bone density and increase bone metabolism, which increase fracture risk after trauma [49]. History of osteoporosis is required, and performing early CT after the trauma has valuable effect in detecting the fracture pattern and the presence of bone fragments in the spinal canal.

The article "Medical Communication Services after Traumatic Spinal Cord Injury" was retracted in 2023. Reasons: signs of a paper mill; suspected computer-generated content; unreliable results or conclusions; concerns about the data.

### 3.4. Surgery and ISP

Laminectomy was found to be ineffective in reducing ISP because it does not affect the pressure between the dura and the swollen spinal cord in chronic SCI, but in some cases with incomplete SCI, ASIA grade C and D, spinal stenosis, or degenerative disease, laminectomy alone can show good outcomes. Adding durotomy to duroplasty can lessen the ISP to less than 20 mm Hg and increase the intradural space, which relieves the blockade of spinal epidural veins and arterioles of cord and prevents CSF leakage. The underlying arachnoid after durotomy becomes pulsatile, intact, and undisturbed. “Trap-door” durotomy allows safer exposure to access the ventral spinal cord with excellent visualization and better evacuation of hematomas, but dural incision of durotomy and duroplasty is a high-risk surgical procedure [11]. Moreover, paralysis after myelotomy can be the result of fault technique through cutting the cord or secondary inflammatory changes [50]. Combined partial myelotomy with radiation therapy showed significant increase in tissue repair than myelotomy alone. Performing myelotomy in the first 24 h is beneficial and can improve the prognosis [51]. A study presented 21 cases with or without intramedullary hemorrhage, and they concluded that durotomy or myelotomy is safe and could reduce secondary injury. However, some cases remained grade A on the ASIA scale after durotomy, but the feeling and sensations obviously improved in most of unimproved patients. Even few cases showed no changes after durotomy, but compared with other procedures, durotomy allows for the best neurological recovery because it has many advantages over other procedures. Durotomy can treat spinal compartment syndrome, decrease ISP, and reduce the edema around intact cord; however, durotomy and duroplasty need a high experience surgeon and high risk at the swollen cord [52]. Current researchers focus on monitoring and predicting SCPP at injury site, which play a critical role in reducing inflammatory process and improve the prognosis.

The article "Medical Communication Services after Traumatic Spinal Cord Injury" was retracted in 2023. Reasons: signs of a paper mill; suspected computer-generated content; unreliable results or conclusions; concerns about the data.

Collected articles include 324 animals that underwent different procedures. Eighty animals underwent myelotomy procedures. Fifty percent showed good outcomes, but 25% showed improvement after myelotomy with anteroposterior plane. Twenty rats with acute SCI underwent myelotomy that showed motor and neurological improvement. Even myelotomy showed improvement, but in some way, it showed negative outcomes by reducing BBB scores. Other studies suggest durotomy as a treatment choice because it treat spinal compartment syndrome, reduces ISP, and leads to better neurological outcomes. Duroplasty limits meningeal fibrosis, decreases scar formation, prevents CSF leakage, and reduces macrophage accumulation, which prevent acumulation of inflamatory process and avoid further injury (Figure 1).

After injury, increasing the pressure around the swollen cord can affect the blood vessels and cause congestion that decreases the blood flow at the injury site. There is limited space around the spinal cord that protects it and allows blood to flow around it. The elasticity feature of the dura can allow flexible space around a healthy spinal cord. After an injury, the swollen cord becomes compressed by the dura, which worsens the situation. Thus, performing durotomy can allow the surgeon to better visualize and evacuate the hematoma to reduce the chances of secondary injury around the swollen cord. The risks associated with durotomy can be avoided depending on the experience of the surgeon and the starting point of the incision. Diffusion tensor imaging (DTI) can show the exact anatomical level of the injury, the severity of the injury, help in classifying the injury severity, and allow direct examination of tissue microstructures. Moreover, DTI identifies the white matter that connect separate parts of the spinal cord. These techniques help to map specific spinal cord regions before surgery and show the severity of the intact cord. Duroplasty can increase the space around the swollen cord, thus improving CSF circulation. Some complications may follow the durotomy with duroplasty, such as CSF leakage, pseudomeningocele, and injured the cord during the procedure, which can be treated by observation or some other intervention depending on the amount of CSF. Observing the situation for a few minutes after duroplasty and before closing the wound can help determine if CSF is leaking out from any site. If it is, it can be managed before closing the wound using fibrin glue or any other method the surgeon decides to employ. If a complication appears postoperatively, and if it affects the cord function or if the patient expresses any complaints, further management may be needed, such as drainage or surgical intervention. Durotomy with duroplasty is the procedure that is used to treat SCI ASIA grades A-C (Figures 2(a) and 2(b)), which can be helpful for treating spinal cord compartment syndrome and improving the clinical or experimental outcomes. Moreover, the physician should consider the patient's bone density, mechanism of the injury, and the bone fragments after the fracture that may affect the dura or worsen the outcome. As mentioned above, ASIA grades A-C need special management; in some cases, the prognosis for laminectomy alone may not be good, depending on the severity of the injury, the length of the swollen cord, and the presence of hematoma. This shows the importance of using another technique (e.g., Laser speckle contrast imaging, Doppler US, or measuring the swollen cord length using a 3D technique) to confirm the situation after laminectomy and to determine if durotomy and duroplasty are required.

The article "Medical Communication Services after Traumatic Spinal Cord Injury" was retracted in 2023. Reasons: signs of a paper mill; suspected computer-generated content; unreliable results or conclusions; concerns about the data.

Early surgical intervention presents better outcomes: surgery within twelve hours of injury can result in better outcomes and avoid further inflammatory process. Additionally, quick understanding and early surgery (durotomy or duroplasty) are essential steps to better prognosis and recovery [53] and shorter hospital stays [54].

The normal physiological ISP range is 2.7–0.5 mm Hg. ISP rises to the range of 4.3–0.8 mm Hg 30 minutes after injury and remains elevated for up to one week. To achieve better long-term prognosis, appropriate early interventions are necessary.

### 3.5. Monitoring ISP and Increasing SCPP

ISP is determined by the size of the CSF space around the cord. Factors that may lower ISP include older age, excess alcohol consumption, nonconus medullaris injury, expansion duroplasty, and less intraoperative bleeding. No MRI factors correlated with ISP or SCPP_opt_. Expansion duroplasty and continuous ISP monitoring by Codman probe is a crucial way to improve patients' prognosis [47]. While monitoring ISP by Codman probe, which has a thinner and longer cable, is a safe technique that appears to enable optimized and individualized spinal cord perfusion [4], patient position is also important because a supine position can increase ISP. A lateral position is better for patients who are being monitored by Codman probe, but a ring-shaped pillow can also be used to support patients in a supine position to avoid increasing ISP. Increases in pressure can cause subacute posttraumatic ascending myelopathy [55]. In some instances, aggravated venous hypertension and/or arterial hypotension at the injury site and equivalent degrees of dural occlusion can cause loss of branch blood flow, which may lead to impaired spinal cord perfusion and can produce additional secondary injury [56].

The article "Medical Communication Services after Traumatic Spinal Cord Injury" was retracted in 2023. Reasons: signs of a paper mill; suspected computer-generated content; unreliable results or conclusions; concerns about the data.

Monitored SCPP by the placement of lumbar subarachnoid drain (LSAD) or visualizing the blood flow at injury site by laser speckle contrast imaging is an essential factor to predict the prognosis and checking the margin of necrosis tissue at injury site.

Increasing SCPP to a level above 50 mm Hg is a strong predictor of improved neurologic recovery [8, 32]. Increased SCPP seems to be linked with enhanced neurological recovery, although monitoring spinal cord perfusion via the MAP's effect on neurological recovery after acute traumatic spinal cord injury is uncertain [57]. Maintaining MAP above 85 mm Hg can improve cord perfusion [7, 28, 58]. However, the relationship between rising motor evoked potential (MEP) and increasing SCPP estimates the damage of the corticospinal tract and predicts function recovery [26]. Lin et al. injected AS-IV medicine intraperitoneal in rat models after SCI through injection, which showed that AS-IV can promote functional recovery [59]. Different methods can detect and calculate the ISP and SCPP, but it needs further study. Different treatment method with different opinion, inserting Codman probe, is safe to monitor ISP for a week; durotomy showed significant improvement in many cases, but adding duroplasty will be better, myelotomy is safe in some patients. Durotomy has different complication, but in many cases, it recovered with neurological improvements. Any procedure to treat the spinal cord has a risk factors and needs experienced surgeon. So visualizing blood flow at injury site, size of the necrosis tissue, anatomical level of the swollen cord, length of the swollen mass, and diameter of the spinal cord at the swollen site can be helpful before and during the treatment period.

### 3.6. Different Factors for Better Outcomes

Rapid diagnosis, time of surgical intervention (laminectomy with durotomy and duroplasty), continued ISP monitoring, placing patients in lateral positions postoperation, maintaining SCPP and ISP, and using special techniques intraoperatively (laser speckle contrast imaging or ultrasound) are strong predictors of prognosis. Using MRI has significant advantages, but sometimes, the initial MRI misses some information [60, 61].

The article "Medical Communication Services after Traumatic Spinal Cord Injury" was retracted in 2023. Reasons: signs of a paper mill; suspected computer-generated content; unreliable results or conclusions; concerns about the data.

Using laser speckle contrast imaging intraoperatively can show blood flow at the injury site, if there is necrosis, and the size of necrosis tissue. These measurements can help predict neurological outcome post injury. It also shows blood flow pulse, which can indicate blood vessel occlusion if the pulse is high/low [34]. Visual inspection of an acutely injured spinal cord can reveal some attributes that are not visible on the initial MRI, and the diameter of the cord can be seen on ultrasonography [12, 29]. To prevent further pressure and injury after the operation, place the patient in a lateral position. There are few limitations in this review: lack of human articles about myelotomy procedure, only few studies compared the durotomy and myelotomy outcomes, and no enough articles mentioning the risk of performing durotomy or myelotomy procedure.

SCPP mainly depends on the MAP and ISP, so maintaining MAP more than 110 and less than 130 with ISP ≤20 mmHg as a standard value to prevent secondary injury and achieve the blood flow in enough amount at the injury site. If SCPP is less than 60 mmHg, it can cause further ischemia, so improving the MAP and keeping the ISP at ≤20 mmHg level can improve the blood flow and avoid ischemia at the injury site. Increasing ISP or decreasing MAP can affect the SCPP value and cause further complications and affect the patient's prognosis. Moreover, checking the patient's history to clarify any reason that influences the MAP affects the SCPP value and worsen the prognosis. The severity of the injury plays a critical role and causes high ISP and low SCPP. ISP is decreased to a suitable value by opening the dura and a CSF pulse around the swollen cord is achieved. The earliest intervention to decrease ISP will show a better outcome. Firstly, ISP needs to be decreased before improving the MAP. Without decreasing ISP ≤20 mmHg, one cannot reach the exact SCPP for a better outcome (Table 3).

## 4. Conclusion

Taking focus on patient history after SCI and cooperating with multidisciplinary team can help to achieve better outcomes. Monitoring ISP and predicting SCPP are critical factors in the treatment of SCI, in addition to early surgical intervention and using proper methods to treat the injury. Data show that the SCPP after the injury was 90–100 mmHg and >60mmHg to avoid ischemia, MAP of 110–130 mmHg, and the mean ISP after an injury is ≤20 mmHg. Severe injury show higher ISP than acute injury. ISP at the injury site is higher than above or below injury site. Using laminectomy alone is not enough to reduce ISP and achieve good prognosis in some cases. Additional durotomy with duroplasty with the removal of necrotic tissues can increase intradural space, decrease ISP, and increase SCPP, which needs to be followed up with a larger randomized, controlled trial to determine if monitoring and SCPP optimization improve outcome. Combination procedure (laminectomy with durotomy and duroplasty) can reduce the ISP below 20 mmHg. Continuous ISP monitoring at the injury site for up to one week is safe. Checking the blood flow to predict the prognosis and the pathophysiology at the injury site is very important during and after the operation to evaluate patients' follow-up recovery and to identify certain pathological changes that are not evident at admission time. Repetitive MRI is essential after 12 hours of initial MRI. DTI can show the severity of injury and the prognosis after the treatment. Lumbar CSF drainage might help to decrease ISP but not enough to improve prognosis.

The article "Medical Communication Services after Traumatic Spinal Cord Injury" was retracted in 2023. Reasons: signs of a paper mill; suspected computer-generated content; unreliable results or conclusions; concerns about the data.

## Figures and Tables

**Figure 1:** Traumatic spinal cord injury. This includes the inflammatory process because of oxidative damage factors, edema, hemorrhage, arterial vasospasm and occlusion, and necrosis tissues at the injury site.

**Figure 2:** (a) Durotomy with duroplasty procedures. A 44-year-old man, remain ASIA grade B before the operation. This patient underwent laminectomy, and CSF pulsation was absent, while after durotomy, the CSF pulsations were recovered, and duroplasty was performed to increase the space around the injured cord. Final follow-up time showed neurological improvements; ASIA grade is C. (b) A 54-year-old man, with ASIA grade A before operation. This patient underwent laminectomy and CSF pulsation was absent, while after durotomy, the CSF pulsations were no recovery, and duroplasty was performed to increase the space around the injuried cord. Final follow-up time (15 months) showed no improvements; ASIA grade remains A.

**Table 1:** Summary of animal studies used, including author and year, number of animals and a short description of the study, and the conclusion achieved.

Reference	Study description	Conclusion
[41]	40 rats, myelotomy	The anteroposterior plane showed significant improvement
[2]	36 rats, laminectomy and durotomy	Increased ISP was maintained by the pial and dural compartments
[35]	24 rats, laminectomy with or without dural repair	Laminectomy does not reduce intraspinal pressure
[36]	72 rats, laminectomy and durotomy ± duroplasty	Functional recovery was better after durotomy and duroplasty
[37]	15 pigs, laminectomy followed by durotomy	Durotomy lowers elevated pressure
[38]	84 rats, laminectomy ± durotomy	Rapid neurological recovery can be better after longitudinal durotomy
[42]	20 rats, myelotomy	Myelotomy has no advantage, and it worsened outcome as shown by reduced BBB scores
[9]	13 pigs, ultrasound was used to visualize the dura and subarachnoid space dimension	Decompression after acute SCI may produce residual cord deformation accompanied by gradual or immediate swelling, causing subarachnoid occlusion
[43]	20 rats, myelotomy	Myelotomy improved motor function and reduced edema
[39]	65 rats, laminectomy ± myelotomy	Myelotomy up to 48 hours after injury can improve the recovery
[44]	81 rats, laminectomy ± myelotomy	Laminectomy plus myelotomy show better outcomes during the postoperation period
[40]	8 dogs, myelotomy ± steroid injection	Myelotomy ± steroid injection did not show significant advantages
[51]	Adult female rats, partial myelotomy ± radiation therapy	Significant increase in tissue repair after myelotomy with radiation therapy

Different procedures were performed in animal studies, where durotomy was the most common procedure, followed by myelotomy. BBB: Basso, Beattie, Bresnahan; SCI: spinal cord injury; ISP: intraspinal pressure.

The article "Medical Communication Services after Traumatic Spinal Cord Injury" was retracted in 2023. Reasons: signs of a paper mill; suspected computer-generated content; unreliable results or conclusions; concerns about the data.

**Table 2:** Summary of the clinical articles used in this review, including author and year, number of patients, treatment method, a brief description of the study, and the conclusion obtained.

Reference	Study description	Conclusion
[11]	1 patient, laminectomy and durotomy	“Trap-door” durotomy is a safe procedure with excellent visualization.
[3]	6 patients, laminectomy and durotomy	Laminectomy and durotomy reduce spinal cord compartment syndrome.
[26]	18 patients, continued ISP monitoring	Monitoring of ISP at the injury site is safe.
[13]	21 patients, laminectomy rather than laminectomy and duroplasty	Adding duroplasty helps decrease ISP and increase SCPP.
[27]	42 patients, laminectomy and ISP monitoring	Continued ISP monitoring is secure and safe for up to one week.
[28]	14 patients, continued SCPP monitoring	Measurement of SCPPopt helps predict prognosis.
[25]	45 patients, laminectomy with durotomy and duroplasty	Reduced ISP or increased SCPP may improve the prognosis posttraumatic spinal cord injury (TSCI).
[8]	1 patient, laminectomy and durotomy	The patient showed no changes.
[29]	8 patients, scaffolds device inserted in the intramedullary cavity	Five patients showed improvement and three remained the same ASIA grade.
[15]	87 patients, laminectomy rather than laminectomy with durotomy	Early intradural microsurgery is safe.
[5]	64 patients, monitoring ISP and SCPP	Expansion duroplasty can increase space around the cord and reduce ISP.
[21]	1 patient, laminectomy and durotomy	Quick diagnosis and rapid evacuation can achieve better neurologic recovery.
[20]	2 patients, laminectomy	The patients showed good recovery.
[12]	1 patient, laminectomy and durotomy	The patient improved remarkably.
[23]	1 patient, laminectomy with durotomy and duroplasty	Good neurological recovery was achieved.
[18]	11 patients, durotomy and 10 patients, myelotomy	Durotomy or myelotomy is safe, and they may also reduce secondary injury.
[17]	17 patients, laminectomy, durotomy, duroplasty	Laminectomy with durotomy and duroplasty inhibit edema and decrease ISP.
[30]	15 patients, lumbar subarachnoid drain (LSAD) for SCPP monitoring	Monitoring SCPP for five days based on LSAD was effective.
[24]	1 patient, partial laminectomies and durotomy	The patient recovered fully with no complications
[16]	1 patient, laminectomy, durotomy, and duroplasty	The patient showed improvement. Double-layer duroplasty might be beneficial to prevent CSF leakage.
[34]	22 patients, laser speckle contrast imaging intraoperatively at the injury site	Acute and severe TSCI yields three patterns of blood flow disturbance at the injury site.
[33]	22 patients, drainage or nondrainage of CSF	Lumbar drainage of CSF was not substantially helpful.
[32]	92 patients, mean arterial pressure (MAP) and CSF pressure were monitored	Maintaining SCPP over 50 mm Hg is a substantial predictor of recovery after SCI.
[19]	30 patients, laminectomy + myelotomy followed by rehabilitation	The procedure showed significant improvement in all the patients. Moreover, rehabilitation for three months is very helpful for the prognosis.
[22]	4 patients, myelotomy	Good prognosis in patients upper limb.

Different procedures were performed in human studies. Studies of different procedures performed in clinical cases, where many patients underwent ISP and SCPP monitoring, and where durotomy was the most common procedure used to treat SCI, followed by durotomy with duroplasty. LSAD: lumbar subarachnoid drain placement; CSF: cerebrospinal fluid; SCPP: spinal cord perfusion pressure; SCI: spinal cord injury; MAP: mean arterial pressure; TSCI: traumatic spinal cord injury; SCPPopt: optimum spinal cord perfusion pressure; AISA: American Spinal Injury Association impairment scale; SCBF: spinal cord blood fusion.

The article "Medical Communication Services after Traumatic Spinal Cord Injury" was retracted in 2023. Reasons: signs of a paper mill; suspected computer-generated content; unreliable results or conclusions; concerns about the data.

**Table 3:** Summary of the data after reviewing the literature, including the conclusion achieved, and a brief description of the conclusion obtained.

Study type	Type of monitoring and intervention	Summary
Animal study	Myelotomy	(1) The anteroposterior plane showed significant improvement (2) Myelotomy improved motor function and reduced edema in some cases (3) Myelotomy has no advantage, and it worsened outcome as shown by reduced BBB scores
	Laminectomy	Laminectomy does not reduce intraspinal pressure
	Durotomy and duroplasty	(1) Functional recovery was better after durotomy and duroplasty (2) Durotomy lowers elevated pressure (3) Rapid neurological recovery can be better after longitudinal durotomy (4) Decompression after acute SCI may produce residual cord deformation accompanied by gradual or immediate swelling, causing subarachnoid occlusion
	ISP	(1) ISP start increasing 30 min after injury and remain elevated up to seven days (2) ISP varied from 8.9 mmHg to 25 mm Hg. These differences are attributable to physiological, anatomical, different species, and severities of injury (3) ISP varied between different species because of differences in physiological, anatomical, and severity of the injury (4) The pial and dural compartments maintained increased ISP

Clinical	Laminectomy, durotomy, and duroplasty	(1) Laminectomy and durotomy reduce spinal cord compartment syndrome (2) “Trap-door” durotomy is a safe procedure with excellent visualization (3) Early intradural microsurgery is safe (4) Quick diagnosis and rapid evacuation can achieve better neurologic recovery (5) Expansion duroplasty can increase space around the cord and reduce ISP (6) Laminectomy with durotomy and duroplasty inhibit edema and decrease ISP (7) Adding duroplasty helps decrease ISP and increase SCPP (8) Double-layer duroplasty might be beneficial to prevent CSF leakage (9) Laminectomy alone cannot reduce the ISP
	CSF drainage	Lumbar drainage of CSF was not substantially helpful
	ISP and SCPP	(1) Monitoring of ISP at the injury site is safe (2) Continued ISP monitoring is secure and safe for up to one week (3) Reduced ISP or increased SCPP may improve the prognosis of posttraumatic spinal cord injury (TSCI) (4) Measurement of SCPPopt (∼90 mm Hg) helps predict prognosis (5) Monitoring SCPP for five days based on LSAD was effective (6) Maintaining SCPP over 60 mm Hg is a substantial predictor of recovery after SCI to avoid ischemia (7) Spinal cord perfusion pressure 90 to 100 mmHg minimized metabolic derangement at the injury site (8) High ISP if >20 mmHg and normal if ≤20 mmHg. In supine position, the patient recovery will be disrupted by high ISP and low SCPP. The supine position should be avoided. A prone position on a ring-shaped pillow can prevent further pressure at the injury site (9) Best recovery when SCPP 90–100 mmHg
	MAP	(1) Maintained MAP between >110 and <120 mm Hg for the first seven days postinjury associated with better neurologic outcome (2) Improving the SCPP through (MAP and CSF pressure) is associated with better neurologic outcome (3) Keeping MAP between 85 and 90 can cause SCPP less than 60, which might cause ischemia

Studies of different procedures performed in humans and animals. LASD: lumbar subarachnoid drain; CSF: cerebrospinal fluid; SCPP: spinal cord perfusion pressure; SCI: spinal cord injury; MAP: mean arterial pressure; TSCI: traumatic spinal cord injury; SCPPopt: optimum spinal cord perfusion pressure; AISA: American Spinal Injury Association impairment scale; SCBF: spinal cord blood fusion; BBB: Basso, Beattie, Bresnahan; ISP: intraspinal pressure.

The article "Medical Communication Services after Traumatic Spinal Cord Injury" was retracted in 2023. Reasons: signs of a paper mill; suspected computer-generated content; unreliable results or conclusions; concerns about the data.

## Data Availability

The data used to support the findings of this study are obtained from collected articles through PubMed, Web of Science, Academia website, and Google Scholar.
